The article "Medical Big Data and Postoperative Nursing of Fracture Patients Based on Cloud Computing" was retracted in 2023. Reasons: suspected computer-generated content; unreliable results or conclusions; concerns about the data; concerns about the results or conclusions.

# Medical Big Data and Postoperative Nursing of Fracture Patients Based on Cloud Computing

**DOI:** 10.1155/2022/4090235

**Published:** 2022-07-11

**Authors:** Li Yan, Yufei Chen, Gao Caixia, Wu Jiangying, Li Xiaoying, Li Zhe

**Affiliations:** ^1^China Medical University, The Fourth Affiliated Hospital of China Medical University, Shenyang, Liaoning 110032, China; ^2^Department of Orthopedics, Air Force Medical Center of PLA Department of Orthopedics, The Fourth Medical Sciences, Beijing 100142, China

## Abstract

Based on the standards for wireless sensor system identification, the sensor node identity OID identification and the management object OID identification in the SNMP MIB are merged, and a management object OID identification coding mechanism for the SNMP-based wireless sensor system is proposed to make the node management system only. The identity, attributes, and multiple entities of the target sensor node in the wireless sensor network can be identified and managed by the node management object OID. The source of abnormal medical big data generally uses two models of multidimensional data and sliding window for detection and verification. First, the sliding window can be used to detect abnormalities. The result is that under this condition, the detection rate of medical big data is more than 95%; the effect is very good, but in different dimensions, the detection rate of four-dimensional data is 2.9% higher than that of a single-dimensional one. On the basis of the ZigBee wireless network, the terminal signal transmission of fracture treatment can be realized. On this basis, combined with the actual needs of fracture treatment, it can be built with its wireless module. The wireless network has a certain basic function. The reform of the nursing system was carried out on the basis of the safety and reliability of the nursing system, the efficiency of the nursing system was improved, and timely and safe nursing services were achieved.

## 1. Introduction

In recent years, with the rapid development of global electronic information technology, especially MEMS, wireless sensor system technology, and wireless communication technology, wireless sensor system technology has also made a breakthrough. A wireless sensor network (WSN) is a collection of independent sensors with the functions of sensing, computing, and communication distributed in a certain area. These sensor nodes are basically low-power memory devices. Wireless sensor networks are widely used in sensing environment, monitoring tasks, control machinery, health care monitoring, industrial monitoring, tracking, and other fields. With the development of global medical computerization, China has also made rapid progress in this field. These big data medical resources have immeasurable value for medical and health information [1]. In particular in the diagnosis, treatment and research of disease have important value. Health care expense management medical big data mainly comes from clinical medicine, disease monitoring, medical research, pharmaceutical companies, expense management, bioinformatics, health care, social networks, etc. Big data promotes the establishment of medical information in China. Technologies related to medical big data have solved some difficulties and problems that cannot be solved before. The future research focus of relevant academic researchers will be on how to make full use of big data technology to solve difficulties [2]. Fracture refers to the complete or partial destruction of the continuity of bone structure, which is more common in children and the elderly, as well as in young and middle-aged people. Usually, some patients have multiple fractures. Through timely and appropriate treatment, most patients can restore their original function, and some patients may have different consequences. Fracture surgery is usually used to repair cartilage lesions, and doctors use arthroscopy to remove the damaged cartilage [3]. Microfracture treatment is a relatively safe and effective method for the treatment of full-thickness cartilage injury of the knee joint. At present, China's clinical nursing practice cannot provide basic nursing, condition monitoring, medication, treatment, communication, and medical care for patients with multiple nursing responsibilities, so as to provide continuous and comprehensive nursing system for patients [4]. The main reason is that when human resources are scarce, nurses will provide treatment for patients and cannot capture the changes of the disease in real time and dynamically. Therefore, it is of great practical significance to improve the development of advanced hospital Internet of things system and related application software and hardware system.

## 2. Related Work

The literature introduces the overall plan design of the nursing system. This section first analyzes the existing problems in the current wireless sensor network node management solution, then introduces the sensor node identification technology and management protocol SNMP used in this solution, and gives the overall system architecture design [5]. Finally, it elaborates the overall scheme design of the system. The literature introduces the design and development of the SNMP manager module on the node management server and realizes the binding of the node management object OID and the SNMP management message and the function of addressing the target gateway by the management object OID; the application in the sensor network gateway is distributed. The management characteristic SNMP proxy agent can realize the management of the sensor node equipment in the large-scale and heterogeneous wireless sensor network of the node deployment and realize the conversion and forwarding of the SNMP management protocol and the function of addressing the target node by the management object OID. Build a node management information database model suitable for wireless sensor networks in the sensor nodes, and implement conventional node management functions [6]. The literature introduces the network architecture of LoRa's wireless self-organizing sensor network, the hardware design of the communication module, and the software design of each module in the overall network. On this basis, a LoRa-based multihop, self-organizing network and rapid test data are built. The wireless self-organizing sensor network was used to do actual tests to verify the stability of the network and the correctness of the data [7]. The literature introduces the LANDMARC positioning system in the RFID positioning algorithm, analyzes some factors that affect the positioning accuracy in the LANDMARC positioning system, and optimizes the selection of reference tags to reduce the error selection rate of the reference tags. Finally, the error correction value is introduced to eliminate the error caused by the RSS. Positioning error is caused by error. After comparing, analyze the advantages of the algorithm proposed in this paper [8]. The literature introduces the design of the overall block diagram of the system and the analysis of key technologies. Combined with the overall framework of the hospital, the system can be divided into three modules: wireless transmission of infusion information, wired transmission of ward call information, and mobile PDA nursing. Show the overall block diagram of the IoT architecture of each module [9]. After checking and analyzing the on-site requirements of the infusion and the security of the call information transmission, it was finally decided that the information collected by the infusion would be transmitted wirelessly through the ZigBee network. The call information on the workstation is transmitted through the CAN bus through the cable, and the PDA handheld system is connected in the form of Wi-Fi [10]. The literature introduces the implementation principle of the classic LANDMARC positioning algorithm in the RFID indoor positioning system and then simulates and analyzes several factors that affect the positioning accuracy of the LANDMARC positioning algorithm and analyzes the areas that can be optimized in the LANDMARC positioning algorithm [11]. Finally, a LANDMARC positioning algorithm based on reference tag selection optimization and error correction value is proposed. The algorithm first reduces the selected error rate and then introduces the error correction value, calculates the error correction value of the reference label most similar to the label to be located, and adds it to the positioning result of the former to obtain the coordinates of the label to be located. The simulation shows that the proposed DISTANCE-LIMIT-LANDMARC algorithm has smaller positioning error and better positioning effect.

## 3. Wireless Sensor System and Medical Big Data Research

### 3.1. Wireless Sensor System Architecture

Each sensor node in the wireless sensor network is composed of a processor module, sensor module, memory, battery, and communication module. The sensor module realizes the function of data acquisition in the covered area; the communication module is mainly for communication and data interaction. The processor module realizes the function of data storage and processing. The hardware structure of wireless sensor network node is shown in Figure 1.

The wireless sensor network mainly includes four parts, as shown in Figure 2, namely, control center, Internet, sink node, and sensor node. Some nodes in the sensor node will act as cluster nodes to manage most of the sensor nodes in the network.

In Figure 2, each cluster node of the network directly manages its subordinate sensor nodes and forms a data link that directly communicates with the sink node. The sink node then transmits the data to the Internet, and the user can obtain the data in front of the terminal equipment of the control center. The design of sensor nodes is not immutable, but the implementation principle is roughly the same; only different processors and communication protocols are used according to different environments and scenarios [12]. When choosing processors, according to the requirements of low power consumption, most of them will choose low-power MCU as the microprocessor. The location of sensor nodes in the network is randomly distributed, but in some application scenarios, it is necessary to know the location of each wireless sensor node. In this way, the data of each sensor node will collect the temperature, humidity, and pressure values and then summarize them and transmit them to the whole network, so that users can consult the data in time.

### 3.2. Key Technologies

#### 3.2.1. Network Protocol

The main function of the network protocol is to make all nodes in the whole link form an interconnected transmission network according to multihop routing. There are two protocols: network layer and data link layer. The network layer also has many shortcomings, such as in the node, storage, and communication, leading to the communication being not smooth, but its operation principle is through information decision management and then control and then perception, acquisition, and transmission process [13]. Due to the objective influence of cost and power consumption, the protocol cannot be relatively complex. At the same time, due to the self-organization and stability of the wireless sensor network, the network protocol needs to have intelligent and dynamic topology, which makes the development of network protocol more difficult.

#### 3.2.2. Topology Control Technology

The main reason why the topology of wireless sensor network is always in a changeable state is the lack of communication ability, coupled with the real-time changes of the external environment, which makes the topology of the whole wireless sensor network always in a changeable state, not fixed. However, a good topology control strategy can avoid these disadvantages perfectly and achieve the effect of high efficiency, energy saving, and cycle improvement.

#### 3.2.3. Data Fusion Technology

Due to the large-scale deployment of wireless sensor networks, the number and density of nodes in the whole network are large, and the similarity is high within a certain range. The large amount of redundant data transmission will lead to the loss of more energy and reduce the life cycle of the whole network [14]. The collection method of basic data and multipath forms the wireless sensor network to a certain extent. Technically, it can reduce the transmission flow and communication to process the data, and it can also use data fusion to process multiple data to improve the security and integrity function.

#### 3.2.4. Time Synchronization Technology

The time synchronization of nodes in the wireless sensor network is an important guarantee for the whole system to work together. NTP and GPS are the common time synchronization mechanisms. The NTP protocol is widely used on the Internet, which is not applicable to networks with unstable structure and less links. GPS has good precision, but the requirements of cost and space environment are high. Therefore, neither of them can be applied in the wireless sensor network well.

#### 3.2.5. Network Security Technology

After the sensor nodes in the wireless sensor network have completed the data monitoring of the target area, the data needs to be processed and transmitted to the user. In this process, the security issues such as various threats and malicious code attacks should be avoided. Therefore, the security problem is the key issue that the whole wireless sensor network needs to pay attention to.

#### 3.2.6. Node Positioning Technology

In order to ensure the accuracy of data, we use randomly distributed sensor nodes. In a specific scenario, the location data of each sensor node is the premise of the existence of the whole wireless sensor network, which is very important to some extent. By using unknown and known data, this process is called node positioning process. Of course, for the present, on the basis of ranging, angle and distance become the main factors in the positioning process.

### 3.3. Medical Big Data Calculation Model

If *s*% of transactions in association rule set *D* contain item set *X*∩*y*, the specific expression of the support degree of association rule is *s*% confidence and support as follows:

(1) $$\begin{array}{c} \text{Supp}\left(X\Rightarrow Y\right)=P\left(X⋃Y\right), \end{array}$$

(2) $$\begin{array}{c} \text{Conf}\left(X\Rightarrow Y\right)=P\left(Y\;|\;X\right). \end{array}$$

When the support and confidence of an association rule are greater than the minimum support threshold min_sup and the minimum confidence threshold min_conf, the association rule is called a strong association rule. The specific conditions are as follows:

(3) $$\begin{array}{c} \text{Supp}\left(X\Rightarrow Y\right)\geq \text{mi}{\text{n}}_{\text{s}}\text{up}, \end{array}$$

(4) $$\begin{array}{c} \text{Conf}\left(X\Rightarrow Y\right)\geq \underset{-}{\min}\text{conf}f. \end{array}$$

Among them, the minimum support threshold and the minimum confidence threshold can be self-defined according to specific applications. When the mined association rules meet these two conditions at the same time, the association rule is valid; otherwise, the association rule is invalid.

Connect *L*_*k*−1_ to itself, if it meets

(5) $$\begin{array}{c} \left(I_{m}\left[1\right]=I_{n}\left[1\right]\right)\&\left(I_{m}\left[2\right]=I_{n}\left[2\right]\right)\cdots \cdots \cdots \left(I_{m}\left[k-1\right]=I_{n}\left[k-1\right]\right)\&\&\left(I_{m}\left[k\right]<I_{n}\left[k\right]\right). \end{array}$$

It is considered that *I*_*m*_ and *I*_*n*_ are connectable. The result of connecting *I*_*m*_ and *I*_*n*_ is

(6) $$\begin{array}{c} \left\{I_{m}\left[1\right],I_{m}\left[2\right],\cdots \cdots ,I_{m}\left[k-1\right],I_{n}\left[k-1\right]\right\}. \end{array}$$

The probability-based interest model is as follows:

(7) $$\begin{array}{c} \text{Int}\left(X\Rightarrow Y\right)=\frac{1-P\left(Y\right)}{\left(1-P\left(X\right)\right)\left(1-P\left(Y\;|\;X\right)\right)}. \end{array}$$

The difference-based interest model is as follows:

(8) $$\begin{array}{c} \text{Int}\left(X\Rightarrow Y\right)=\frac{\text{Conf}\left(X\Rightarrow Y\right)-\text{Supp}\left(Y\right)}{\max\left(\text{Conf}\left(X\Rightarrow Y\right),\text{Supp}\left(Y\right)\right)}. \end{array}$$

The interest degree model based on correlation is as follows:

(9) $$\begin{array}{c} \text{Int}\left(X\Rightarrow Y\right)=\frac{\text{Supp}\left(X\cup Y\right)}{\text{Supp}\left(X\right)\text{Supp}\left(Y\right)}. \end{array}$$

Among them,

(10) $$\begin{array}{c} \text{Supp}\left(X\cup Y\right)=\frac{\text{Count}\left(X\cup Y\right)}{N}, \end{array}$$

(11) $$\begin{array}{c} \text{Supp}\left(X\right)=\frac{\text{Count}\left(X\right)}{N}, \end{array}$$

(12) $$\begin{array}{c} \text{Supp}\left(Y\right)=\frac{\text{Count}\left(Y\right)}{N}. \end{array}$$

The degree of interest is defined as

(13) $$\begin{array}{c} \text{Int}\left(X\Rightarrow Y\right)=P\left(X\right)\left[P\left(Y\;|\;X\right)\log\left(\frac{P\left(Y\;|\;X\right)}{P\left(Y\right)}\right)+\left(1-P\left(Y\;|\;X\right)\right)\log\left(\frac{1-P\left(\left.Y\right|\right.}{1-P\left(Y\right)}\right)\right]. \end{array}$$

The influence-based interest model is as follows:

(14) $$\begin{array}{c} \text{Int}\left(X⟹Y\right)=\log\frac{\text{Conf}\left(X\Rightarrow Y\right)/\text{Conf}\left(X\Rightarrow \overset{¯}{Y}\right)}{\text{Supp}\left(Y\right)/\text{Sup}\left(\overset{¯}{Y}\right)}=\log\left(\frac{N-\text{Count}\left(X\right)}{\text{Count}\left(X\right)-\text{Count}\left(X\cup Y\right)}\times \frac{\text{Count}\left(X\cup Y\right)}{\text{Count}\left(Y\right)}\right). \end{array}$$

The interest degree model is as follows:

(15) $$\begin{array}{c} \text{Int}\left(X⟹Y\right)=\text{Conf}\left(X\Rightarrow Y\right)-\text{Conf}\left(\bar{X}\Rightarrow Y\right)=\frac{P\left(X⋃Y\right)}{P\left(X\right)}-\frac{P\left(\overset{⟶}{X}\cup Y\right)}{P\left(\overset{¯}{X}\right)}=\frac{P\left(X\cup Y\right)-P\left(X\right)P\left(Y\right)}{P\left(X\right)\left[1-P\left(X\right)\right]}, \end{array}$$

(16) $$\begin{array}{c} \text{Conf}\left(X\Rightarrow \overset{¯}{Y}\right)=\frac{N-\text{Count}\left(X\cup Y\right)}{\text{Count}\left(X\right)}, \end{array}$$

(17) $$\begin{array}{c} \text{Supp}\left(Y\right)=\text{Count}\left(Y\right)/N, \end{array}$$

(18) $$\begin{array}{c} \text{Supp}\left(\overset{¯}{Y}\right)=\frac{N-\text{Count}\left(Y\right)}{N}. \end{array}$$

There are 25 cases of both coughing and flu, 10 cases of coughing but no flu, 15 cases of coughing but no flu, and 80 cases of coughing and flu.

The calculation is as follows: the degree of support for a patient with a cough and the possibility of flu is

(19) $$\begin{array}{c} \text{Supp}\left(A\Rightarrow B\right)=P\left(A\cup B\right)=\frac{25}{120}=20.8\%. \end{array}$$

The above conclusions can be drawn:

(20) $$\begin{array}{c} P\left(\frac{B}{B}\;|\;A\right)<P\left(\frac{B}{\overset{¯}{B}}\right). \end{array}$$

And if the interest degree model of this article is introduced, the calculation can get

(21) $$\begin{array}{c} \text{Int}\left(A\Rightarrow B\right)=\text{Conf}\left(A\Rightarrow B\right)-\text{Conf}\left(\overset{¯}{A}\Rightarrow B\right)=\frac{25}{35}-\frac{80}{85}=-0.227. \end{array}$$

It can be seen that

(22) $$\begin{array}{c} \text{Int}\left(A\Rightarrow B\right)<0\&\&\left|\text{Int}\left(A\Rightarrow B\right)\right|<\underset{-}{\min}\mathrm{int}, \end{array}$$

(23) $$\begin{array}{c} H_{m}=\left\{\text{rule file of }L_{k}\text{ has }m\text{ items}\right\}, \end{array}$$

(24) $$\begin{array}{c} \left(I_{m}\left[1\right]=I_{n}\left[1\right]\right)\wedge \left(I_{m}\left[2\right]=I_{n}\left[2\right]\right)\wedge \cdots \wedge \left(I_{m}\left[k-2\right]=I_{n}\left[k-2\right]\right), \end{array}$$

(25) $$\begin{array}{c} L_{k}=\left\{c\in C_{k}\;|\;\text{ c}.\text{count}\geq \underset{-}{\min}\mathrm{supp}\right\}. \end{array}$$

It is meaningful to improve and optimize the classic Apriori algorithm by introducing the degree of interest.

### 3.4. Algorithm Simulation

Research on optimization of the Apriori algorithm is based on cloud computing and medical big data.  Figure 3 shows the comparison of the traditional Apriori algorithm. The minimum interest threshold of the improved algorithm is 0.3, and the minimum interest threshold of the improved algorithm is 0.45, which is under different minimum support thresholds [15]. Obviously, the improved algorithm will degrade fewer association rules at the same minimum support threshold and integrate the number of degraded association rules in inverse proportion to the minimum interest threshold. A reasonable minimum interest threshold can be set through experience to exclude association rules that users are not interested in.

A total of 6 experiments were performed on the set size, and the experimental results are shown in Table 1.

According to the above experimental results, we can draw a line graph of the serial parallel algorithm, as shown in Figure 4.

The above experimental results show that the improved MapReduce-based Apriori algorithm based on the Hadoop platform has great advantages in processing big data.

It can be seen from the figure that after 37 MB, the serial algorithm consumes a lot of memory and then cannot complete the associated mining. Although it will gradually become larger with the scale, there will be a turning point at 37 M, resulting in insufficient memory. However, since the Hadoop platform runs in a pseudo-parallel mode, the tasks of parallel algorithms need to be exchanged. Therefore, when the data is small, it is more advantageous to use serial algorithms.

A total of 4 experiments were carried out for different transaction set sizes, and the experimental results are shown in Table 2.

According to the above experimental results, draw a line chart, as shown in Figure 5.

This section aims at system simulation. At the beginning, we show how to create a simulated Hadoop platform and introduce the three distribution modes of the Hadoop platform. The first is simulation, and the premise is carried out in pseudo-parallel distributed mode; the second is to determine the size of the data set, and this method is performed in the distributed mode; the third is to analyze the final conclusion in time. The Apriori algorithm is more suitable because it is faster and more accurate when processing big data.

## 4. Design and Application of the Nursing System after Fracture Treatment

### 4.1. System Architecture Design

The clinical medical infusion monitoring system based on the Internet of things technology consists of three parts: the infusion information acquisition terminal, the ward call system, and the PDA handheld terminal. The drip irrigation information terminal is mainly responsible for collecting the drip irrigation rate, setting an appropriate drip irrigation rate value according to the patient's condition and issuing an alarm when the actual drip irrigation rate deviates from the normal value or the drip irrigation ends [16]. The ward call system warns patients who need to press a button in an emergency. The PDA handheld terminal system allows medical staff to obtain basic patient information by scanning the QR code on the patient's wristband when visiting the ward. Each part uses a different wireless communication method, and each part has an IoT control unit [17]. The lower part of the control unit is the lower computer responsible for collecting and processing various information and data, and the upper part of the control unit is the upper computer responsible for collecting data. Data information is stored and displayed through the remote client terminal.

The overall structure block diagram of this system is shown in Figure 6.

### 4.2. Monitoring Terminal Design

#### 4.2.1. Methods of Obtaining Patient Information

Intravenous drip is a routine clinical treatment for hospitalized patients, but it is characterized by tedious and repetitive tasks. Intravenous infusion patients use different types of drugs, the types of drugs will be updated quickly, and the nurse cannot be notified of new drugs in time, which may be a risk factor for intravenous surgery [18]. At the same time, as patients become more and more self-sufficient, this requires safer and more effective hospital infusion operations. At that time, a new wireless injection system based on RFID technology came into being.

The wireless infusion system based on RFID technology uses a handheld mobile PDA to scan the patient's wristband and infusion tag, so that health care professionals can obtain correct basic patient and medication information. Whether it is a doctor or a patient, the injection will start after observation and confirmation [19]. At the same time, the mobile care system will actively record various information to prevent accidents, especially to further confirm the operability and time to achieve safety effects. After the infusion is completed, the system will print out the various statuses of the infusion process as soon as possible, so that the effect of checking at any time can be achieved. The system uses mobile phones and barcode technology on many connections to change and improve the way the hospital operates its original process connections, further enhancing safety awareness, which can force medical staff to pay more attention to service quality and standards.

#### 4.2.2. Design of Droplet Monitoring Scheme

In addition to an infusion pump, there are various infusion monitoring equipment in the market, and many methods are used. However, the technology used for liquid monitoring uses the photoelectric principle to detect liquid level. It is mainly used to determine whether the infusion has been completed [20]. Install the grating in the fixed position of the injection bottle. When the liquid level in the infusion bottle drops to the position of optoelectronic sensor, the light sensor uses the reflection and refraction of light to determine whether the infusion is completed. There are also major restrictions because it is not suitable for drug packaging when used. The liquid is monitored using the conductivity of the metal electrode [21]. Insert two metal electrodes into the sample tube or bottle. According to the different conductivities of air and liquid and metal electrode, different resistance values are used to record the injection. This process will pollute the liquid, so it cannot be used for intravenous injection in clinical medicine.

#### 4.2.3. Design of the Infusion Monitoring Terminal

The infusion information acquisition terminal consists of two parts: infusion information acquisition unit and drop information processing control unit. The infusion information acquisition unit includes external infrared detection module, single chip system, liquid crystal display, droplet speed confirmation button, emergency call button, and wireless transmission module [22]. Its main function is to measure and display the droplet velocity, and the patient can manually control the alarm injection process abnormality or completion of injection.

#### 4.2.4. Scheme Design of the Ward Call System

The station call system is a comprehensive system project, which should be considered in terms of its function, performance, cost, and the latest technology application. Because of this demand, it is best to use CAN bus technology to develop many integrated intelligent medical call systems, which have functions such as hospital bed calls, toilet calls, and corridor screen displays [23]. Each site in the site is regarded as a node, and the signals collected by the site nodes are transmitted to the main site call signal processing controller through two lines of CAN_H and CAN_L serial differential transmission.

### 4.3. Communication Module Design

As far as the current society is concerned, wireless communication technology has become a hot target in various fields. In this case, the global health care industry tends to use wireless local area networks.

In terms of wireless networking modes in this project, the following modes are used:

Networking based on ZigBee technology: the site area is relatively large, because ZigBee technology is even suitable for wireless data transmission in a small area. In a large and relatively complex building environment, the loss rate of radio signals should be high [24]. Using additional equipment methods to improve the ability to send and receive data will not be able to solve the problem of radio signal conflicts and the high possibility of errors, and it will not be possible to establish a large-scale sensor network throughout the hospital. In addition, ZigBee terminals have higher energy requirements because they must always transmit signals and use wired power mode.

Wi-Fi-based network: a PDA handheld device is a very mature technology of Wi-Fi. It does not need to send and receive data, and exchange data with the advanced management system wirelessly and exchange data through Wi-Fi. Analyzing the problem can ensure stable bedside patient monitoring data transmission.

Network based on wired CAN bus transmission technology: the word call system uses a CAN bus to realize data transmission. This is mainly to ensure reliable transmission while ensuring security, but it has the disadvantages of poor system scalability and the need for verbatim input [25]. Based on the above content, this project will take the construction of a single ward as an example to build a very low power consumption, simple operation, and an expandable clinical medical monitoring system based on RFID technology.

The built-in positioning system consists of three types of wireless nodes: coordinator, positioning node, and reference node. The coordinator is the core of the entire system and is responsible for building and managing the entire network [26]. The coordinator sends the RSS value and coordinates received from the positioning node to the computer through the serial USB interface, and then, the corresponding higher-level computer software calculates the graph. The reference node must provide the RSSI value of the positioning node and its own location information. Each reference node returns the received RSSI value of the positioning node and its own position information to the positioning node, and the positioning node returns RSS and the like from each reference node [27].

### 4.4. Information Management System Design

The main function of the clinical medical information management system is to monitor the infusion status of patients in real time, respond to the needs of patients in a timely manner, understand the conditions and needs of each ward, and scientifically manage the entire ward. The work efficiency has been improved, so the ward has been improved. And the capacity of health professionals has improved.

The information management system is based on the current three-tier architecture model, which is mainly divided into data, business, and application levels. The basic structure is shown in Figure 7.

The business function of the system requires data support. The data is collected from other databases, and the company uses ETL tools combined with API (application programming interface) services to classify, aggregate, and appraise the data. Unified verification, processing, calculation, storage and management of data, formulating unified access and output standards according to business needs, creating a big data layer, and putting each business function into actual operation make them more efficient and accurate.

This section introduces the basic knowledge of indoor wireless positioning technology, LoRa-based wireless ad hoc network, and RFID-based indoor positioning algorithm optimization through the previous sections as the theoretical support of this section. Part of the RFID positioning optimization model and algorithm proposed in Section 4 is verified in the LoRa-based wireless ad hoc sensor network. The feasibility and stability of the LoRa-based wireless self-organizing sensor network and the superiority of the proposed RFID-based indoor positioning optimization algorithm are verified through experimental verification, data collection, and comparative analysis.

### 4.5. Software Parameter Setting

The setting of the data frame format is to determine whether the data transmitted during the communication process is valid, so as to ensure that the data of the sender and the receiver are correct.

There are two types of wireless transmission data frames in the infusion monitoring system:

The working status data frame of the infusion monitor is shown in Table 3.

The response data frame of the infusion monitor is shown in Table 4.

At the same time, the corresponding codes are given for the working state of the equipment in the wireless infusion monitoring system. The corresponding codes of working status information are shown in Table 5.

## 5. Conclusion

At present, the medical industry is always people's livelihood issue, which is related to the rise and fall of everyone, even a family. In this case, how to be transparent, convenient, and information-based has always been the goal of human pursuit and also the fundamental way to win the popular support. With the development of science and technology, big data has become a hot research object. How to use the modern technology of big data to apply in the medical industry has become the focus of attention. In view of the huge amount of medical big data, the traditional collection methods have been unable to meet the growing needs. Cloud computing can be said to be the best solution. With the help of the cloud platform of health care, it collects, processes, and stores the relevant data, so that health care workers and patients can view the information they need anytime and anywhere, to suit the remedy to the case or to carry out targeted operation. This is also the trend of the future. The potential information value of medical big data is endless. Of course, the difficulty in front of us is how to use it reasonably, which is the most important. This paper proposes data mining technology and association rules to solve this problem. Through professional computing and platform application, combined with multidimensional data and sliding window model, the multimode data streaming mode in the wireless sensor network can be obtained. It can evaluate the degree of variance of data points through calculation and further identify the source of abnormal data, so as to solve the problem pertinently, so as to improve the algorithm and reach the accurate standard. Therefore, the final results show that this method is our ideal type and can achieve our expected goal.

## Figures and Tables

**Figure 1:** Hardware structure of the wireless sensor network node.

**Figure 2:** Architecture of the wireless sensor network.

**Figure 3:** Comparison of the number of association rule mining between the improved Apriori algorithm and the classic algorithm.

**Figure 4:** Performance line chart of the serial parallel algorithm.

**Figure 5:** Line chart of parallel algorithm performance in fully distributed mode.

**Figure 6:** The overall structure block diagram of the system.

**Figure 7:** Nursing monitoring system architecture diagram.

**Table 1:** Performance comparison of serial and parallel algorithms.

Transaction set size (KB)	Number of association rules	Serial algorithm mining time (s)	Parallel algorithm mining time (s)
1310	14684	33	131
2440	15005	71	215
4670	15010	129	278
9240	15084	264	395
18500	14977	605	621
37500	14893	N/A	1150

**Table 2:** Performance simulation of the parallel algorithm in fully distributed mode.

Transaction set size (MB)	Number of blocks	Mining time (s)
298	6	3142
596	12	6312
910	19	9543
1217	25	12386

**Table 3:** Data frame of the transfusion monitor working state.

Initial identification	Department code	Ward code	Bed number	Equipment code	Status code	Information number	Check digit
%	Section	Bedroom	Bed	Device	State	In£	%

**Table 4:** Nursing monitor response data frame.

Initial identification	Bed code	Status code	Information number	Check code	Initial identification
%	Bed_NO	State	Inf	%	%

**Table 5:** Corresponding code of transfusion monitor working status information.

Boot up	0F10	Error	0F30	Start infusion	0F50	End of infusion	0F70
Normal detection	0F20	Insufficient charge	0F40	User call	0F60	Shut down	0F80

## Data Availability

The data used to support the findings of this study are available from the corresponding author upon request.

## References

[1] Lai Y.-C., Hsiao L.-Y., Chen H.-J., Lai C.-N., Lin J.-W. (2013). A novel query tree protocol with bit tracking in RFID tag identification. *IEEE Transactions on Mobile Computing*.

[2] Hossain M. A., Sarkar N. I. (2018). A distributed multichannel MAC protocol for rendezvous establishment in cognitive radio ad hoc networks. *Ad Hoc Network*.

[3] Lopez D. A., Rojas C. A., Zapata D. F., Trujillo E. R. (2018). Designing a MAC algorithm for equitable spectrum allocation in cognitive radio wireless networks. *Wireless Personal Communications*.

[4] Kadam S., Prabhu D., Rathi N., Chaki P., Kasbekar G. S. (2019). Exploiting group structure in MAC protocol design for multichannel ad hoc cognitive radio networks. *IEEE Transactions on Vehicular Technology*.

[5] Feng P., Bai Y., Huang J., Wang W., Gu Y., Liu S. (2019). CogMOR-MAC: a cognitive multi-channel opportunistic reservation MAC for multi-UAVs ad hoc networks. *Computer Communications*.

[6] Liu Y., Yu R., Pan M., Zhang Y., Xie S. (2017). SD-MAC: spectrum database-driven MAC protocol for cognitive machine-to-machine networks. *IEEE Transactions on Vehicular Technology*.

[7] Qureshi F. F., Iqbal R., Asghar M. N. (2017). Energy efficient wireless communication technique based on cognitive radio for Internet of things. *Journal of Network and Computer Applications*.

[8] Zikria Y. B., Ishmanov F., Afzal M. K., Kim S. W., Nam S. Y., Yu H. (2017). Opportunistic channel selection MAC protocol for cognitive radio ad hoc sensor networks in the Internet of things. *Sustainable Computing: Informatics and Systems*.

[9] Miao G., Azari A., Hwang T. (2016). E2-MAC: energy efficient medium access for massive M2M communications. *IEEE Transactions on Communications*.

[10] Saad W., El-Feshawy S. A., Shokair M., Dessouky M. I. (2018). Optimised approach based on hybrid MAC protocol for M2M networks. *IET Network*.

[11] Verma P. K., Verma R., Prakash A. (2016). Machine-to-machine (M2M) communications: a survey. *Journal of Network and Computer Applications*.

[12] Wang H., Fapojuwo A. O. (2017). A survey of enabling technologies of low power and long range machine-to-machine communications. *IEEE Communications Surveys and Tutorials*.

[13] Cisco VNI Mobile (2017). Cisco visual networking index: global mobile data traffic forecast update, 2016–2021 white paper.

[14] Hong S., Brand J., Choi J. I. (2014). Applications of self-interference cancellation in 5g and beyond. *IEEE Communications Magazine*.

[15] Sarret M. G., Berardinelli G., Mahmood N. H., Mogensen P. Can full duplex boost throughput and delay of 5g ultra-dense small cell networks?.

[16] Song L., Li Y., Han Z. (2015). Resource allocation in full-duplex communications for future wireless networks. *IEEE Wireless Communications*.

[17] Marasevic J., Zhou J., Krishnaswamy H., Zhong Y., Zussman G. (2017). Resource allocation and rate gains in practical full-duplex systems. *IEEE/ACM Transactions on Networking (TON)*.

[18] Sun Y., Ng D. W. K., Ding Z., Schober R. (2017). Optimal joint power and subcarrier allocation for full-duplex multicarrier non-orthogonal multiple access systems. *IEEE Transactions on Communications*.

[19] Cirik A. C., Rikkinen K., Latva-aho M. Joint subcarrier and power allocation for sum-rate maximization in OFDMA full-duplex systems.

[20] da Silva J. B., Xu Y., Fodor G., Fischione C. Distributed spectral efficiency maximization in full-duplex cellular networks.

[21] Goyal S., Liu P., Panwar S. S., DiFazio R. A., Yang R., Bala E. (2015). Full duplex cellular systems: will doubling interference prevent doubling capacity?. *IEEE Communications Magazine*.

[22] Nam C., Joo C., Bahk S. (2015). Joint subcarrier assignment and power allocation in full-duplex ofdma networks. *IEEE Transactions on Wireless Communications*.

[23] Tehrani P., Lahouti F., Zorzi M. Resource allocation in OFDMA networks with half-duplex and imperfect full-duplex users.

[24] Di B., Bayat S., Song L., Li Y., Han Z. (2016). Joint user pairing, subchannel, and power allocation in full-duplex multi-user ofdma networks. *IEEE Transactions on Wireless Communications*.

[25] Nam C., Joo C., Bahk S. Radio resource allocation with inter-node interference in full-duplex OFDMA networks.

[26] Osterb O. Scheduling and capacity estimation in LTE. In Proceedings of the 23rd international teletraffic congress, ITC’11.

[27] Park T., Shin O.-S., Lee K. B. Proportional fair scheduling for wireless communication with multiple transmit and receive antennas.

